# An innovative microcoring technology: A novel approach to acne scar treatment

**DOI:** 10.1111/srt.13545

**Published:** 2024-01-04

**Authors:** Hyo‐Sang Ahn, Soo‐Kyung Kim, Ruri Pamela, Pei‐Hsuan Lu, Vanravi Vachatimanont, Ardhiah Iswanda Putri, Henry Tanojo, Kyu‐Ho Yi

**Affiliations:** ^1^ Division in Anatomy and Developmental Biology, Department of Oral Biology Human Identification Research Institute, BK21 FOUR Project, Yonsei University College of Dentistry Seoul South Korea; ^2^ Pharmaceutical Industry Department, Graduate School Chung‐Ang University Seoul South Korea; ^3^ CELV Dermatology Clinic Jakarta Indonesia; ^4^ Medical Director of Haute Age Medicine Clinic Taipei Taiwan; ^5^ iSKY Center Bangkok Thailand; ^6^ Rejuva Clinic Surabaya Indonesia; ^7^ Melania Clinic Surabaya Indonesia; ^8^ Maylin Clinic (Apgujeong) Seoul South Korea

**Keywords:** acne scar, minimally invasive, rotational fractional resection, scar treatment

## Abstract

**Background:**

Acne scars present a complex challenge in dermatology and cosmetics, despite advancements in technological interventions such as fractional lasers, microneedling, and surgical procedures. Effective treatment remains elusive for many individuals.

**Objective:**

This study aims to evaluate the efficacy of rotational fractional resection using 1 mm diameter rotating scalpels as a primary treatment for icepick and boxcar scars on the cheeks and glabella region.

**Methods:**

Three patients with acne scars underwent a single treatment session of rotational fractional resection. Evaluation occurred at the 2‐month post‐treatment mark to assess improvements in scar appearance and potential skin‐related side effects.

**Results:**

Following the treatment, significant improvements were observed in the targeted acne scars. Notable enhancements were noted without major skin‐related adverse effects, except for minor suture marks.

**Conclusion:**

The outcomes of this study underscore the potential of rotational fractional resection as an innovative and effective approach in treating acne scars. This single‐session cosmetic procedure shows promise in yielding lasting and quantifiable results, offering a hopeful solution for individuals seeking comprehensive acne scar treatment.

## 1 INTRODUCTION

Acne scars on the face pose a common cosmetic concern, characterized by distinct and complex topographic changes in the skin surface. The multifaceted nature of facial scars, each with its unique characteristics, makes their management a challenging endeavor. Various clinical methods, including chemical peels, fractional lasers, microneedling, and energy‐based devices, have been employed to address facial scars, yet they often fall short in delivering sustainable results in scar treatment. Fractional ablative laser therapy, utilizing CO2 or Er:YAG lasers, has emerged as an effective approach for facial scar management. These techniques leverage a controlled wound‐healing process to transform scar tissue into healthy tissue. However, the high‐energy lasers used in this treatment lead to extended recovery periods and potential side effects, such as burns and hyperpigmentation, limiting their applicability to certain scar types. Additionally, there is a risk of collateral tissue damage due to the heat generated by laser devices.^1^

Microcoring needles have been suggested as an innovative approach to address grafting scars by targeting the removal of fibrous bands and the skin tightening resulting from the elimination of the dermal‐epidermal column.^2^ Coring needles, akin to fractional ablative lasers, can eliminate multiple small, full‐thickness skin columns without the photothermal harm associated with lasers. The rapid rotation of a microneedle is recognized for its ability to reduce unintended damage while precisely ablating the intended tissue. Due to the absence of extensive thermal injury to surrounding tissues, the recovery time and post‐inflammatory hyperpigmentation can be managed. In this research, microcoring techniques were applied to assess the outcomes in three clinical cases involving acne scars.

## 2 MATERIALS AND METHODS

In our procedures, we employed the microcoring system integrated with the N‐Derm platform from N‐finders, Korea, Inc. This system utilizes 1 mm diameter rotating scalpels to perform resection of scars in the cheek and glabellar region (Figure 1). The study strictly followed the principles outlined in the Declaration of Helsinki, including its subsequent revisions, and was conducted in full accordance with the pertinent ethical guidelines. Prior to the procedures, informed consent was duly obtained from all participants.

**FIGURE 1:** Illustrates a schematic representation of the microcoring system, where the controlled rotation of a micro‐needle (A) leads to the specific removal of the target tissue (B) through the ablation of the dermal‐epidermal column.

### 2.1 Clinical experiment

Exclusion criteria for this study encompassed a history of mechanical allergies, significant medical conditions, or any facial treatments, surgical or nonsurgical, conducted within the preceding 6 months. All patients received comprehensive explanations regarding the study's objectives and procedures. Patients who had developed hypotrophic scars due to steroid injections were also excluded from the study. Three participants, consisting of one female and two males aged 32, 46, and 49 years, respectively, were involved in the treatment (Video S1). Topical anesthesia, in the form of lidocaine cream, was applied for 30 min before the procedures. For local anesthesia at the scarring site, dental lidocaine with epinephrine was administered. The procedure was executed using a handheld rotational micro‐coring scalpel with a single punch, with the needle's depth being manually adjusted. A 1 mm inner diameter coring needle was employed to create full‐thickness skin holes, ranging from the epidermis to the superficial subcutaneous fat, with the assistance of jeweler forceps to eliminate any remaining debris.

Following the creation of the hole using the jeweler's forceps, the residual tissue was subsequently removed (Figure 2). Closure of the wound resulting from rotational micro‐coring was accomplished using 7‐0 nylon sutures. Following the procedure, prophylactic oral cefalexin (500 mg, three times daily for 5 days) was administered, and the resected sites were closed with sutures, coupled with the application of a stretched elastic adhesive dressing to facilitate wound healing. After a week, the compressive dressings were removed, and patients attended follow‐up appointments on the day of the procedure, at 7 days, 1 month, and 2 months postoperatively. At the 2‐month follow‐up, patient satisfaction was assessed using a self‐report questionnaire, with options for “very satisfied,” “satisfied,” “disappointed,” or “very disappointed,” along with inquiries about any treatment‐related side effects, such as persistent pain, folliculitis, erythema, edema, hyperpigmentation, or hypopigmentation. In addition to the self‐questionnaire, two dermatologists evaluated bleeding (ranging from none to severe) and examined the healing progress, looking for signs of ecchymosis, purpura, fluid accumulation, hyperpigmentation, hypopigmentation, roughness, dryness, inflammation, erythema, crusting, scarring, and any adverse events.

**FIGURE 2:** A 1 mm inner diameter coring needle was employed to create full‐thickness skin holes, multiple for larger scars, ranging from the epidermis to the superficial subcutaneous fat (A), with the assistance of jeweler forceps to eliminate any remaining debris (B).

## 3 RESULTS

No unfavorable incidents, including severe side effects, were documented in any of the clinical trials. Pain experienced in the facial skin during the procedure was quantified using a Visual Analog Scale (VAS) score, with scores of 3, 2, and 3 recorded during the procedure itself. Post‐procedure VAS scores stood at 2, 2, and 2 on day 1 and reduced to 0, 0, and 0 on days 7 and 4, respectively. In the course of treatment, two patients encountered minor bleeding, while one experienced moderate bleeding. Examination of visible scars in photographs taken after 2 months of treatment revealed grading by two dermatologists as ranging from “severe” to “mild” and one dermatologist assessing them as ranging from “mild” to “almost clear.” The self‐questionnaires completed by the three patients indicated that two were highly satisfied, and one was satisfied (Figure 3). Notably, no patient reported enduring pain, folliculitis, erythema, edema, hyperpigmentation, or hypopigmentation.

**FIGURE 3:** A 46‐year‐old man displaying a boxcar scar (A) underwent the microcoring procedure on the right side of his cheek. The microcoring system employed was the N‐Derm platform by N‐finders, Korea, Inc, utilizing 1 mm rotating scalpels to excise the boxcar scar, followed by suturing (B). Twelve weeks after the treatment (C).

## 4 DISCUSSION

While scars themselves may not pose medical issues, they are a prominent cosmetic concern for numerous individuals. The three primary clinical factors contributing to the development of acne scars include the severity of the initial acne lesion, the individual's skin type and genetics, and the efficacy of early scar management and treatment. These factors, combined with the unique characteristics of each scar, can make the effective management of acne scars a multifaceted challenge. The study of Liu et al. aimed to assess global acne scar prevalence and risk factors in acne patients. Analyzing 37 studies involving 24,649 individuals, we found a 47% prevalence of acne scars. Significant risk factors identified were male gender, positive family history of acne, and increased acne severity. Early intervention and effective therapy in managing acne are crucial to reduce acne scarring based on these findings.^3^ The study of Lofti et al. investigates the efficacy of a combined treatment, utilizing radiofrequency‐assisted subcision and polycaprolactone‐based dermal fillers, for managing atrophic post‐acne scars, demonstrating significant improvements in various acne lesion types but suggesting the need for larger randomized clinical trials for more conclusive findings.^4^

Acne scars encompass several distinct types, including atrophic scars such as icepick, boxcar, and rolling scars, which create varying degrees of depressions in the skin (Figure 4). Hypertrophic scars appear raised and thickened but remain within the original injury boundary, while keloid scars extend beyond it. Post‐inflammatory hyperpigmentation (PIH) results in discolored marks post‐acne lesion healing, and erythematous scars manifest as temporary red or purplish spots. The choice of treatment for these acne scars depends on their type and severity, necessitating professional evaluation by a dermatologist for appropriate treatment selection.

**FIGURE 4:** Acne scars encompass several distinct types, including atrophic scars such as icepick (A), rolling (B), and boxcar (C) scars, which create varying degrees of depressions in the skin. For the Microcoring system, icepick, and boxcar are ideal targets for the treatment.

Moreover, as acne scars are visible dermatological conditions, they represent chronic issues that have both physical and psychological impacts on a substantial number of patients.^5^ The repercussions often extend to a reduction in quality of life and can lead to psychological challenges such as depression and social avoidance.^6^ Various treatments, including chemical peels, nonablative and ablative lasers, as well as fractional lasers, have been employed for scar management. Nevertheless, the majority of these procedures have yielded unsatisfactory clinical results and come with a range of drawbacks, including procedural discomfort, extended recovery periods, and a heightened occurrence of adverse events.

Past research has indicated that fractional lasers exhibit favorable clinical effectiveness in addressing acne scars; nonetheless, these lasers may inadvertently lead to epidermal damage, including burns, and precise adjustments of the radiofrequency thermal zones' depth can be challenging.^7^, ^8^ These constraints are anticipated to be surmounted with the introduction of the recently developed microcoring device.^2^, ^9^

In the initial pig study, microcoring was employed with the objective of skin tightening. The utilization of a coring needle for mechanical skin removal proved to be highly effective in achieving this desired outcome.^10^, ^11^ Following the removal of 10% of the skin through microcoring, the treated area exhibited a reduction of 9%.^11^ Histological analysis of the areas treated with microcoring showed elevated fibroblast activity and collagen production.^10^ An enzyme‐linked immunosorbent assay (ELISA) demonstrated an 89% rise in collagen levels 3 months following the treatment.^10^

Pozner and colleagues conducted a similar assessment of skin tightening in human subjects, and their conclusion was that the procedure is safe and well‐received, demonstrating positive effects on skin rejuvenation. Initial observations included skin tightening and enhanced skin thickness.^9^

In an earlier investigation, Dayan employed a microcoring system to address skin laxity in the submental fat pad and enhance neck rejuvenation for a group of 31 patients. The majority of patients experienced an improvement of at least one grade in skin laxity and lipodystrophy as evaluated by the investigator. A total of 84% expressed satisfaction with the appearance of their neck and jawline, and a noteworthy 97% were inclined to recommend the procedure to others.^2^

An important constraint in this study is the small sample size, consisting of only three participants, which may constrain the broader applicability of the results. Additionally, while stitch scars post‐treatment were not observed in this study, it is imperative to acknowledge the possibility of their occurrence. The potential occurrence of stitch scars post‐microcoring treatment, which may persist after the procedure.

Within the realm of skin tightening, microcoring represents a relatively recent innovation. This technique involves the removal of skin using hollow needles to prevent the formation of scar tissue. This article marks the initial exploration of scar treatment in three clinical cases. It's important to note that the study's primary constraint is its limited sample size. However, the procedure was found to be well‐tolerated, with minimal pain and bleeding both during and after treatment, and the associated outcomes were deemed insignificant. The method has demonstrated safety and a favorable healing profile. Further research and application of this innovative approach should be extended to include conditions like focal vitiligo, tattoo removal, and nevus treatment.

## CONFLICT OF INTEREST STATEMENT

The authors have all considered the conflict of interest statement included in “Author Guidelines.” To the best of our knowledge, no aspect of the authors’ current personal or professional life might significantly affect the views presented on this manuscript. The authors declare no conflicts of interest.

## Supporting information

Supplement Video 1. The dental lidocaine with epinephrine was applied locally at the scarring site, and a handheld rotational micro‐coring scalpel with a single punch was utilized to manually adjust the needle's depth and create full‐thickness skin holes using a 1 mm inner diameter coring needle, assisted by jeweler forceps for debris removal.

## Data Availability

The data that support the findings of this study are available from the corresponding author upon reasonable request.
